# The Application of Public Art Design Based on Digital Technology in Urban Landscape Environmental Monitoring

This article has been retracted.

**DOI:** 10.1155/2022/7882943

**Published:** 2022-10-12

**Authors:** Lingfeng Xie, Junling Zhou, Kuan Liu

**Affiliations:** ^1^College of Fine Arts, Guangdong Polytechnic Normal University, Gaungzhou, Gaungdong, 510665, China; ^2^Faculty of Innovation and Design, City University of Macau, Macau 999078, China; ^3^State Key Lab of Subtropical Building Science, South China University of Technology, Gaungzhou, Gaungdong, 510640, China; ^4^Pelli Clarke & Partners, New Haven, CT 06510, USA

## Abstract

Public art (PA) is a powerful tool for enhancing the environment in public spaces since it not only relieves the oppression caused by urban architecture but also enhances and beautifies urban public spaces. As DT (digital technology) develops so quickly nowadays, it offers PA significant technological assistance to achieve new functions, and changes in modern people's aesthetic preferences and psychological makeup also present new demands for PA. This essay explores the use of PA design in the creation of urban landscapes from the viewpoint of DT. In order to do this, this paper suggests a method for measuring the environmental impact of urban landscapes that combines landscape measurement and semantic assessment. Full-connection algorithm and greedy algorithm are introduced to identify urban functional types with high-dimensional characteristics for the boundary tree classification model of high-dimensional feature classification. The findings indicate that the public service area's producer and user accuracy are, respectively, 0.8783 and 0.7833. It offers a fresh concept for the identification of urban functional zones while solving the issues of low identification efficiency and poor accuracy.

## 1. Introduction

With the growth of PA (public art), more and more people are starting to pay attention to how it works and how it expresses itself, constantly adding new force and elements to the works and bringing to light for more people the possibility of expressing emotions and acquiring cultural inheritance through PA. Modern city PA landscape is helpful for uplifting the living sentiments of city dwellers and can, to some extent, enhance the economic advantages of the city. New technology included into PA's design will emphasise the interactive nature of the works, improve public interaction, and express the cultural spirit in line with the contemporary aesthetic context. In general, strong PA works can be produced as long as there are good concepts for them and they are actively supported by the audience and numerous artists.

PA in urban landscape is an indispensable node in urban landscape, and it is a diversified landscape space construction art with postmodernism artistic character, which includes not only the construction of things in space but also the construction of culture in space. In urban construction, PA did not rise for urban construction at first but was a special activity to meet the needs of cities in a certain era [1]. However, in today's PA construction, there are some phenomena that are contrary to art and public spirit. Taking the urban development and construction out of context, misjudging, and tending to political purposes make most PA become visual rubbish. Without the support of culture, our artistic design will have no life, and our design will be pale and powerless. In urban landscape art, the artistic expression form of “super graphic art” is used to reflect and retain urban culture, instead of wantonly pursuing visual impact [2, 3] and enjoyment. Under the influence of DT (digitization technology), the interactivity of urban PA has changed from the original interaction between people and works of art itself to deeper interaction, and its connotation has changed. This is the problem that this paper focuses on.

Early art is often regarded as elegant art and the art of the rich, and it is difficult for ordinary people to feel the charm of art. PA makes art go from studios and exhibition halls to the public. It can be expressed by sculpture, installation, mural painting, and even other audio-visual arts, such as drama, film, dance, singing, environmental art, multimedia image art, and even avant-garde experimental art such as earth art, performance art, and concept art [4]. The evolution of PA has a strong connection to people's daily lives, and its creative meaning is becoming more closely associated with people's interests in life, which is widely embraced by everyday people. Although the inventive raw materials used to create PA items are from commonplace sources, their meaning is in line with consumer tastes. Urban culture is the culmination of long-term urban growth and the image of urban spiritual civilisation. Landscape PA is a crucial component of urban development since it is a way of passing down urban culture. In the context of graphic art theory, landscape architecture, and PA studies, the abstract analysis of landscape architecture employing DT as the visual communication medium has significant research value.

The innovation of this paper is mainly reflected in the following aspects:

1. Based on the existing technical means, this paper discusses various creative techniques of urban PA landscape interactive design under the digital background, seeks the possibility of combining DT with other art forms, and explores the possible role and increasingly important position of interactive urban PA in the future human life
2. The boundary tree classification model is introduced to formalise the characteristics of urban landscape and spatiotemporal themes, and the automatic identification model of urban functional areas is constructed in light of the fact that the existing research lacks the characteristics of urban landscape to depict urban functions and does not thoroughly consider its spatiotemporal factors and attribute characteristics

There are five chapters in this paper. The following list summarises the important points and research for each chapter: Section 1 presents the research's historical context.  Section 2 primarily introduces the relevant studies on the development of urban landscapes. The PA design mode is presented in Section 3 as a method for creating urban landscapes. The performance of the model examined in this research is validated in Section 4.  Section 5 serves as the epilogue.

## 2. Related Work

### 2.1. Development of PA

PA has special significance in modern urban construction. It is the breaking, reorganization, and innovation of cultural resources and represents the explicit and intuitive cultural values of a country or a city. Many countries have implemented various policies and bills that are beneficial to the development of PA, such as percentage art bill, public cultural policy, and the establishment of art community, to promote the values guided by PA.

Wu and Li think that human beings are about to enter the era of entertainment economy, and the entertainment factor will become an important value-added activity of products and services and the key to market segmentation. No matter what consumers buy, they are looking for the entertainment component [5]. Chen has also done intake research on the new concept of virtual technology and the relationship between human perception, perception, cognition, and motor control ability [6]. Habib and others pointed out that the power problem in PA must be faced squarely by analyzing the dialectical relationship between ancient art and power and further pointed out that PA not only involves art, aesthetics, and technology but also is a social problem. The crux of PA lies in the solution of social problems [7]. Bai et al. took the course and concept of contemporary PA as the research object, made extensive and specific research on the development of contemporary PA, made clear thinking and answers to the opportunities and challenges faced by contemporary PA in China, and put forward their own academic opinions and behavioral propositions [8].

Roehrdanz and others pay more attention to the current society. Artistic works can lead people's spiritual thoughts and lead people out of difficulties. PA not only promotes and develops regional culture but also has a good influence on the construction of tourist cities and the promotion of urban economy [9]. Xiao et al. build the space system of humanistic activities, build the city brand, and highlight the charm of the city [10]. Baouche et al. conducted in-depth research on digital PA and interactive thinking through multidisciplinary research such as art and technology, aesthetics and sociology, PA and new media art, traditional sculpture techniques and digital virtual technology, psychology, and cognition [11].

### 2.2. Research on Urban Landscape Construction

The most common PA work in urban landscape is urban sculpture, which not only has the form of sculpture in appearance but also contains profound artistic connotation with specific regional characteristics. Besides humanistic elements, urban landscape PA also contains cultural expressions of spiritual level, that is, the expression of urban regional environment, the expression of urban history and culture, the expression of urban image and individual characteristics, etc. The expression of the environment provides people with an opportunity to know the city.

Di et al. evaluated the form and theme of PA from the perspective of theoretical criticism and discussed the city's inclusiveness of art form and art [12] in view of the inclusion or exclusion of art. Hai et al. discussed PA products shaped by differences of different classes, races, cultures, regions, and ages from the perspectives of art, space, and identity and analyzed the contradictory problems in social practice to illustrate the interference of problems in reality [13]. Yang et al., through the analysis and research of the literature, obtained that their achievements mainly focused on the development and construction of the physical environment of the waterfront and the publicity of the waterfront [14]. Nuo et al. put forward the development principles, models, legislation, and policies of waterfront areas and separately discussed the landscape juice design methods of waterfront areas [15].

In the theoretical research of urban open space, Ito and others think that open space is a subsystem of urban space system, public property of people, and a space place and environment that is open to the public, allows the public to enter, has certain public facilities, and serves various public activities and social life in the city [16]. Hu and Li used computer three-dimensional graphics method to analyze the visual impact and put forward a quantitative evaluation index of the openness of building exterior space [17]. Qiao et al. made a comprehensive review on the research of urban surface openness, pointing out that the calculation results of urban surface openness are unreasonable at some local points, and the research of urban surface openness should pay more attention to the regional average [18]. Wessels et al. constructed an automatic classification method of urban land use by describing the spatial distribution of buildings, which provided an effective reference for urban function identification based on urban landscape [19]. Robert et al. explored the influence of different spatial locations and places on residents' psychology, such as subjective cognition of happiness, depression, boredom, and affluence [20].

## 3. Methodology

### 3.1. Morphological Analysis of Urban Landscape Elements

The quality of urban environment and landscape PA complement each other and influence each other. Good public landscape affects the cultural heritage of the city and the beautification of the urban environment, while the environmental quality of the city affects the cultural and historical heritage in PA's creation. Therefore, PA should be combined with the environmental characteristics of surrounding areas in the design process, instead of being isolated in a certain environment. With the increasing number of public space art works, artists prefer specific time and place when creating works, and artists are less and less fond of their works being fixed by firmness and place; that is to say, they have given up the pursuit of permanence of PA. Minimalism abandons symbols and symbols, creating a pure abstract form that dispels any emotion and vitality. Pop art's living objects are not only depicting themes but also creating materials. These artistic skills can often enrich the visual expression of artistic modeling, thus endowing PA's works with new vitality.

The various elements in the urban landscape can also be called a form. In essence, the shape of various elements is the three-dimensional shape of the three-dimensional space, and the points, lines, surfaces, and bodies in the form are also relative. Among the buildings in the landscape, a building can be regarded as a point, but when compared with a car, a building is a body. The continuity of points can form a dotted line, and the synthesis of points can form a virtual surface. Although the dotted line and imaginary surface composed of dots are not as clear and firm as the solid line and the solid surface, they are more beautiful in rhythm and rhythm. The wall in space, the floor of enclosed space, the wall and ceiling, the opening of doors and windows in space enclosure, the outline of architectural form, and the monomer form in space.

Sculpture occupies a very important position in urban culture, often showing the authoritative environment and culture, vivid images of styles, and allusions. The unique aesthetic significance permeates into citizens' lives, which makes sculptures in urban public spaces get more and more attention from people with the promotion of urban status and become business cards of cities. The sculpture of public space in the city is the real mapping of people's life in the city, the space carrier of the historical imprint and cultural connotation of the whole city, and the primary manifestation of successfully embodying the urban spirit. The unique aesthetic significance permeates into the life of the city, which makes the sculpture in the public space of the city get more and more attention with the commission of the city status. The reflection of the spiritual life of the city people represents the image of the city.

Uncertain water quality model research has increased in recent years. To properly and thoroughly comprehend and master the changing process of the water environment and comprehend the essence of water environment changes, it is helpful to conduct research and use mathematical models of uncertain water quality. The aquatic environment is a complicated system with many unknowable variables. The main sources of model uncertainty in water quality simulations are the unpredictability of pollutant discharge and river background value. The study of uncertain water quality models is therefore cutting edge and a hot topic in the field of water quality modeling today and in the future. It has significant theoretical and practical implications. At the moment, research on water environment problems that are uncertain both domestically and internationally mostly focuses on the methods and theories of uncertainty that are most frequently employed, such as artificial neural networks, stochastic theory, grey theory, and fuzzy theory. In this paper, an uncertain water quality model is studied using neural networks.  Figure 1 depicts the study of unknown factors in the aquatic environment.

Because neural network is based on data, it can learn and train to master the internal change rules of the system, instead of using mathematical equations to express the relationship between input and output, and its application is simple and convenient, so it is very suitable for dealing with nonlinear water environment problems. Make the analysis and simulation process of water quality more reasonable, improve the prediction accuracy, and enhance the ability to deal with nonlinear problems. The prediction results of an example show that the model is insensitive to the selection of initial values, has good convergence and prediction accuracy, and is suitable for practical engineering applications [14].

The research of uncertain water quality model is a common means to improve and understand various uncertain factors in water environment. According to the assumption, the results of past *n* measurements are taken as the input elements of neural network, and the built-in neural network time-delay uncertain water quality model is

(1) $$\begin{array}{c} u\frac{{dC}_{t}}{dx}=-{kC}_{t}+f\left(C_{t-1},C_{t-2},\cdots ,C_{t-n}\right), \end{array}$$

where *C*_*t*_ is the concentration of a pollutant in the river section at time *t*, mg/L; *u* is the longitudinal flow velocity of the river reach, m/s; *x* is the flow distance from the section to the sewage outlet, m; and *f*(*C*_*t*−1_, *C*_*t*−2_, ⋯, *C*_*t*−*n*_) is a neural network function.

The fitness function *E*_*u*_ is constructed to determine the approximation degree of the function, and each parameter is formed into a parameter set *γ* = (*k*, *a*_*i*_, *w*_*ij*_, *θ*_*j*_). The purpose of optimization is to find the best $\tilde{\gamma }$ and make $E_{u}=J\left(\tilde{\gamma }\right)=\min J\left(\gamma \right)$. For comparison with the deterministic water quality model, the fitness function is selected as follows:

(2) $$\begin{array}{c} E_{q}=\overset{3}{\underset{i=1}{\sum }}\overset{4}{\underset{j=1}{\sum }}\frac{\left|C_{ij}-C_{ij}^{\prime }\right|}{C_{ij}}. \end{array}$$

After the radiant brightness value *L*_*λ*_ is calculated in the first step, the ground brightness temperature can be calculated according to Planck formula, or the ground brightness temperature value can be calculated by using the following deformation formula:

(3) $$\begin{array}{c} T_{d}=\frac{K_{2}}{\ln\left(1+\left(K_{1}/L_{\lambda }\right)\right)}, \end{array}$$

where *T*_*d*_ is the ground brightness temperature (unit: K), *L*_*λ*_ is the radiant brightness temperature, and *K*_1_, *K*_2_ is the correction coefficient, respectively.

There are great differences in boundary length and internal area between irregular patches and standard patches, which can be expressed by the ratio of the actual length of patch boundary to the circumference of the same area. The higher the ratio, the more complex and longer the patch shape, and the more obvious its directivity. The calculation formula is as follows:

(4) $$\begin{array}{c} \text{Shapeindex}=\frac{P}{2\sqrt{\pi A}}, \end{array}$$

where *P* is the perimeter of the visible area and *A* is the area of the visible area.

If the shape index is large, it means that the visible space is complex in shape and blocked in different directions, so the directivity of the openness is obvious. If the shape index is small, the visible space is simple.

### 3.2. PA Design in Urban Landscape Construction

The age of digital art is bringing art and science closer together, and technology is having an effect on all aspects of art. As a result, the existing form of art is significantly impacted by the change in media. The three fundamental types of art have always been painting, sculpture, and architecture. Digital art is not a pure technology under the humanistic restrictions of art; rather, it is an expression of ideas and thoughts. DT offers a variety of practical service means and ways, frees people's hands from difficult and repetitive manual labour, and expands the area available for artistic creation to use schemes and approaches. The most distinctive aspect of digital art is interactive art. Through a variety of technical ways, artists can first interact with intelligent machines before having their works communicate with the audience. They may do their work directly in accordance with the audience's understanding, or they may deduce other tricks in accordance with the protocols. This type of contact may also be reflected in indirect absence and direct presence.

There are flowers, trees, waterfalls, rivers, bridges, and fountains in the external space of the city. These elements not only have their own noumenon functions but also carry the local customs, culture, and historical connotations, which provide a certain foundation for PA's creation. The emergence of digital media technology has greatly enriched the expression forms of PA's creation. Digital controlled lighting technology, digital auxiliary technology, and digital interactive technology have greatly expanded people's imagination. Publicity is the main feature emphasized by PA's landscape design, but it can only be realized through interaction with society, the public, and space. Only when its methods and concepts can be discussed in the field of sociology can it become an art science. From the perspective of cultural themes, there are thematic PA, landscape PA, historical and cultural PA, recreational PA, and ecological PA. This will help to increase the public's interest and participation in PA and make it immersed in PA works all over the world. Watching these arts is like traveling around the world.

It may be claimed that DT is now a way of life for modern folks. It focuses on the everyday life of the subject matter, the technicalization of production, the virtualization of influence, the philosophization of ideas, and the diversification of skills and portrays people's perspectives on life, art, and the world in a cutting-edge, frivolous, and sometimes boring way against the backdrop of the digital age. A new PA power is communicated through the flexible display of intangible material on tangible carriers. Its development is inextricably linked to economic growth, consumer culture's emergence, the diversification of artistic development, and the popularity of artistic expression. It blends in with the surroundings of the location being displayed, and as time and place change, so does the meaning of the object.

Three-dimensional creation is to make it flat in three-dimensional space, which constitutes a new design feature of “super plane art.” The decoration design on the surface of the building makes the whole building look like a huge decorative painting, weakening the feeling of three-dimensional. For example, the sudden appearance of huge color pictures in squares or street corners will give people a new visual experience in urban life where buildings coexist, which also provides opportunities for information transmission. People's consciousness has inertial thinking, so even if we remove some elements from the object form, it still cannot affect our perception system's cognition of the overall shape of the object elements. Let art and cultural knowledge be closer to life and enrich people's thoughts, feelings, and cultural cognition, so as to create a green activity place full of cultural and artistic breath for that public through design, and at the same time, art can make the charm of culture shine and bring people closer to each other's communication and interaction.

Regional division is the first condition for identifying urban functional areas, and it is also an important issue in the study of variable area units in geography [15]. In order to integrate landscape measurement and semantic measurement features and solve the contradiction between “high-dimensional classification features” and “low-dimensional classification model” of urban functional types, this paper adopts the boundary tree classification model for high-dimensional feature classification, introduces the full connection algorithm and greedy algorithm, and realizes the identification of urban functional areas by calculating the maximum boundary between each urban functional type under high-dimensional features.

The boundary *M* of urban function type *C*_*j*_ is calculated as follows:

(5) $$\begin{array}{c} \left(\beta_{0},\beta \right)=\arg\max\left(C_{j}\right),\text{where}Y_{j}\left(\beta_{0}+\underset{i}{\sum }\beta_{i}y_{ij}\right)\geq C_{j}, \end{array}$$

where *β*_0_, *β* is the constant and weighted variable for calculating urban functional characteristics *y*_*ij*_ and *Y*_*j*_ is the classification state of urban functional types.

Check the precision of the urban functional regions' identification results. Utilize quantitative indicators to assess the accuracy of the identification findings based on the confusion matrix, taking into account the types of functional areas and the overall identification accuracy. By using the Kappa coefficient method, urban functional zones are identified.

(6) $$\begin{array}{c} K=\frac{P_{o}-P_{e}}{1-P_{e}}. \end{array}$$

*P*_*o*_ is the ratio of the correctly classified number of each function type to the total number of samples, and *P*_*e*_ is the ratio of the product of the actual number of each function type and the classified number of samples to the square of the total number of samples.

The realization of the three-dimensional openness model suggested in this paper can be generally separated into two steps in accordance with the conceptual model indicated above. As shown in Figure 2, the first step is to determine the obstacle points that block the viewpoint for a specific viewpoint in all directions. The second step is to examine the spatial distribution of the obstacle points using the various indexes indicated above.

Scan the dividing points along the line of sight, obtain the topographic elevation value of the dividing points of the line of sight, and compare the interpolated elevation with the line of sight elevation to judge its visibility. Repeat the fourth and fifth steps for the sight lines with different horizontal and vertical angles until the obstacle points in all directions are obtained. The terrain elevation value is obtained by interpolation, and the openness information in urban space is comprehensively and deeply analyzed and mined by various quantitative statistical methods.

Openness refers to the deviation degree between the geometric center of the projection of a three-dimensional visual sphere on the horizontal plane and the viewpoint. In statistics, skewness is a parameter that describes the characteristics of data distribution. It measures the asymmetry of geographic data distribution and depicts the deviation centered on the central value. The calculation formula is as follows:

(7) $$\begin{array}{c} \text{Skewness}=\sqrt{{\left(x_{v}-x_{o}\right)}^{2}+{\left(y_{v}-y_{o}\right)}^{2}}, \end{array}$$

where (*x*_*v*_ − *y*_*v*_) is the coordinate of the geometric center of the visible area and (*x*_*o*_ − *y*_*o*_) is the coordinate of the viewpoint. If the degree of open deviation is large, it means that the viewpoint is blocked seriously in some continuous or similar directions, while it is blocked slightly in other directions, and the visual space as a whole tends to some directions.

As the distribution of thermal environment of remote sensing images in the same area and different time phases cannot be directly compared, the normalization method is used to classify the surface temperature, and the calculation formula is as follows:

(8) $$\begin{array}{c} N_{i}=\frac{T_{i}-T_{\min}}{T_{\max}-T_{\min}}, \end{array}$$

where *N*_*i*_ refers to the normalized surface temperature value of the *i*th pixel; *T*_*i*_ is the surface temperature value of the *i*th pixel; and *T*_min_, *T*_max_ is the minimum and maximum of the surface temperature in the image.

This study uses a hierarchical clustering method to group urban functional themes based on how similar they are to one another in order to extract the measurable characteristics of urban functional semantics. The DB (Davies-Bouldin) index is chosen as a result, and the better the clustering effect, the lower the DB index. The DB index computation formula is

(9) $$\begin{array}{c} \text{DB}=\frac{1}{N}\overset{N}{\underset{i=1}{\sum }}\underset{j\neq i}{\max}\left(\frac{S_{i}+S_{j}}{d_{TWED}\left(\theta_{c1},\theta_{c2}\right)}\right), \end{array}$$

where *N* is the number of clusters, *S*_*i*_, *S*_*j*_ is the standard deviation of the distribution probability of the *i*th and *j*th text topics, and *c*1, *c*2 are two different clustering results.

Landscape index is the most commonly used method to study landscape ecology. Different landscape indexes are used to describe the landscape pattern, which makes the change process more intuitive [13]. The expression of SHDI (Shannon's Diversity Index) is as follows:

(10) $$\begin{array}{c} \text{SHDI}=-\overset{m}{\underset{i=1}{\sum }}\left(P_{i}\right)\times \log_{2}\left(P_{i}\right), \end{array}$$

where *P*_*i*_ is the proportion of the *i*-type landscape elements in the total landscape area and *m* is the number of patch types. The closer SHDI is to 0, the whole landscape is composed of a patch. The larger the SHDI, the more balanced the distribution of landscape types.

## 4. Experiment and Results

Generally speaking, a complete interactive system of urban PA needs comprehensive consideration of three factors, namely, urban public space, urban PA works, and the main body of urban PA. In interactive city PA, interaction plays a guiding role. In the creation of interactive city PA, it is also a bridge between works and audiences. According to the characteristics of interactive city PA, such as publicity, interaction, aesthetics, and sociality, artists should consider four important design elements, namely, modeling elements, sensory elements, emotional elements, and functional elements.

The research data of this paper include road network data, electronic map data, points of interest, public comments, and data which can be obtained free of charge from all sources of geographic data and land use planning data. By calculating the spatiotemporal themes of urban functions, the distribution probability of 30 themes in 24 time intervals is shown in Figure 3. The distribution probability range of each topic is [0, 1].

The distribution probability of Theme 10 is the highest at around 5 am and 15 pm, and the distribution probability at other times is relatively small, which is consistent with the residential function represented by this theme. Therefore, the model of urban functional area identification based on landscape measurement and semantic measurement has the highest accuracy, followed by the model based on semantic measurement, and the model based on landscape measurement has poor identification results. Through the similarity evaluation of landscape index, the screening of urban landscape features is realized.

According to the method discussed in this paper, the accuracy of the identification model of urban functional areas is verified. The identification accuracy of residential areas, commercial areas, industrial areas, and public service areas is shown in Table 1.

The producer precision and user precision of the public service area are, respectively, 0.6435 and 0.6829 in the results of urban functional area identification based on landscape measurement. The producer precision and user precision of the public service area are 0.8783 and 0.7833, respectively, in the findings of urban functional area identification integrating landscape measurement and semantic measurement. As a result, the model used to identify urban functional areas has high identification accuracy for each urban functional region and integrates landscape measurement and semantic measurement.

A sample area was chosen for each land use type in the study region, and the center point was chosen as the perspective. The quantitative indices of three-dimensional openness of each viewpoint were then calculated in order to analyze the variations in surface openness under various land use types. The findings of the calculation of the viewpoint's three-dimensional openness characteristic index at the center of each sample area are displayed in Table 2.

It can be seen that when the viewpoint is located in residential areas and commercial areas, the height-width ratio of the ladder is obviously higher than that of other land use types. This is because residential areas and commercial areas are densely built, the viewpoint is close to the horizontal distance of buildings, and the building height is large, so the visual landscape is very compact. The former obstacle point does not block the latter obstacle point obviously, and the visual space in the vertical direction is obviously hierarchical, which is easy to divide.

Figures 4 and 5 show that the residential area has the largest variation in viewpoint fluctuation frequency and that the maximum height visible in various horizontal directions changes frequently, reflecting the characteristics of the viewpoint's visual space. The skyline is also rich and vivid, though patchy. Due to the significant height differences between the buildings in the public service area, where the viewpoint is located, the frequency of fluctuations is largest. Experience has shown that there is a correlation between surface temperature and the normalized difference vegetation index [15, 16].  Figure 6 depicts the study area's linear relationship between surface temperature and normalized difference vegetation index as well as the association between urban heat island and normalized difference vegetation index [17].

It can be concluded that the higher the vegetation normalization index, the lower the surface temperature, while the lower the vegetation normalization index, the higher the surface temperature. There is no such negative correlation between normalized difference vegetation index of water body and surface temperature, because the temperature of water body itself is relatively low and the amount of vegetation in water is small, so the above relationship is not suitable for water body. Through rational planning and layout, increasing urban green space area is still one of the effective ways to alleviate the heat island effect of city.

As the natural bioremediation is a process of completely relying on nature, it is far from enough for most polluted water bodies whose ecology has been destroyed, and artificial bioremediation technology must be adopted. There are mainly in situ bioremediation technology and ex situ bioremediation technology. The hydraulic conditions and water pollution characteristics of small and medium-sized urban rivers determine the necessity and importance of applying aeration and oxygenation technology to control river pollution.

The established water quality model of landscape river is used to predict the water quality after the hydrodynamic conditions are improved. The comparison between the predicted results of COD_Cr_ concentration in the river after hydrodynamic conditions is shown in Figure 7.

From the above research, it can be seen that after doubling the hydrodynamic force of the river, the quality of landscape river water has significantly improved. Therefore, improving the hydrodynamic condition is an effective way to improve the water quality. However, due to the constraints of the implementation cost and equipment maintenance of enhancing river hydrodynamic, how to effectively apply this principle needs further research.

## 5. Conclusion

The modern PA landscape of the city is a harmonious and unified system of nature and society. PA landscape is not only a simple decoration in urban landscape but also a new creation of urban culture. Under the background of DT, the interactive design of urban PA has its corresponding principles and elements, as well as its realization ways and methods, which together constitute an independent system. Many digital interactive systems have successfully become cultural landmarks of local cities and achieved great success. The full combination of DT and PA is the inevitable development of technology, and it is also the general trend. The form of its involvement in PA creation has developed from the traditional auxiliary type to the leading type. The urban functional area identification method based on landscape measurement and semantic measurement proposed in this paper shows that the producer precision and user precision of public service areas are 0.8783 and 0.7833, respectively. This method improves the efficiency of urban functional area identification and realizes the automation of functional identification of different cities.

## Figures and Tables

**Figure 1:** Analysis process of uncertain factors in water environment.

**Figure 2:** Flow chart of realizing the three-dimensional openness model.

**Figure 3:** Time distribution probability of urban functional spatiotemporal themes.

**Figure 4:** Located in the skyline of the viewpoint residential area.

**Figure 5:** The viewpoint is located in the skyline of the public service area.

**Figure 6:** Relationship between surface temperature and normalized difference vegetation index.

**Figure 7:** Comparison between the COD_Cr_ value of the predicted section after improved hydrodynamic force and the measured value before.

**Table 1:** Accuracy verification of identification results of urban functional areas.

Domain	Landscape measurement	Semantic measurement	Fusion model
Residential area			
Producer precision	0.6435	0.7298	0.7742
User accuracy	0.6829	0.4422	0.9067
Public service area			
Producer precision	0.6024	0.6866	0.8783
User accuracy	0.4491	0.6129	0.7833
Commercial areas			
Producer precision	0.645	0.624	0.713
User accuracy	0.6364	0.6068	0.8081
Industrial area			
Producer precision	0.7181	0.7591	0.7799
User accuracy	0.6696	0.4091	0.7445

**Table 2:** Three-dimensional openness characteristics of viewpoint located in different land use types.

Sample area type	Obstacle step number	Step height-width ratio	Fluctuation frequency	Fluctuation frequency
Residential area	3.795	1.0411	0.1612	12.0865
Public service area	3.0781	0.496	0.0844	15.1729
Commercial areas	2.7884	1.2551	0.1169	13.283
Industrial area	2.649	0.619	0.1278	14.943
Reserved land	3.6637	0.4787	0.1584	1.7076
Public green area	2.5013	0.3378	0.183	2.5352

## Data Availability

The data used to support the findings of this study are available from the corresponding author upon request.
